This article has been retracted.

# Effect of nHA-Coated Femoral Stem Prosthesis Combined with Platelet-Rich Plasma in Hemi Hip Replacement of Femoral Neck Fracture in the Elderly

**DOI:** 10.1155/2022/9089084

**Published:** 2022-08-10

**Authors:** Lu Yang, Dabin Wu, Tongsheng Liu, Guozheng Fang

**Affiliations:** Department of Orthopaedics, Shanghai Baoshan Luodian Hospital, Shanghai 201908, China

## Abstract

**Purpose:**

This study investigated the efficacy of nanohydroxyapatite- (nHA-) coated biological prosthesis combined with platelet-rich plasma (PRP) in hemi hip replacement of femoral neck fracture (FNF) in the elderly.

**Methods:**

From September 2018 to September 2021, 102 elderly patients with FNF treated in our hospital were chosen and divided into two groups according to different intervention methods. Fifty-one patients in the bone cement group were treated with bone cement prosthesis, and the rest 51 patients in the observation group were treated with nHA biological prosthesis combined with PRP in hemi hip replacement. In order to explore the osteogenic effect of nHA and PRP, osteoblasts were cultured.

**Results:**

It was found that nHA and PRP could both effectively promote the proliferation of osteoblasts and improve their mineralization ability, especially when used in combination. In the course of clinical therapy, we found that the use of biological prosthesis combined with PRP could effectively reduce the level of serum procollagen type I carboxy terminal peptide (PICP) and better improve the levels of bone alkaline phosphatase (BALP) and bone Gla protein (BGP), so as to reduce the bone conversion rate and promote the formation of new bone around the prosthesis. In addition, no significant difference was found in intraoperative bleeding, operation time, hospital stay, 48 h drainage volume, partial weight-bearing time, and complete weight-bearing time between two groups. Otherwise, the use of biological prosthesis could effectively avoid the occurrence of adverse reactions such as bone cement crisis and fracture around femoral prosthesis, so as to better restore the hip function and improve patients' life quality.

**Conclusions:**

Therefore, in hemi hip replacement of FNF in the elderly, nHA biological prosthesis combined with PRP can effectively promote the formation of new bone around the prosthesis stem, so as to obtain good initial stability, enable patients to carry out early weight-bearing exercise, and effectively avoid adverse reactions caused by bone cement prosthesis, thus improving patients' hip function and life quality.

## 1. Introduction

With the aggravation of social aging, due to osteoporosis, the elderly are very prone to fractures due to falls, collisions, and other reasons in the process of daily life, of which hip fractures account for about 50%, and most of them are femoral neck fracture (FNF) [1]. According to statistics, by 2050, the proportion of FNF in systemic fractures will increase from 3.6% to 7%, and most of them are the elderly [2]. FNF is also known as dead fracture in the elderly, and if timely and effective therapy cannot be given, it is very easy to be complicated with a variety of adverse complications because of prolonged bed rest, such as accumulated pneumonia and bedsore, which will cause a heavy economic and spiritual burden to patients and their families [3]. At present, except for patients who cannot tolerate the operation and have obvious surgical contraindications, surgical therapy is recommended for the vast majority of displaced FNF in the elderly [4], so as to restore patients' weight-bearing ability as soon as possible, thus reducing the complications caused by long-term bed rest. With the progress and development of medical technology, hip arthroplasty has become an important method for FNF therapy in the elderly. Compared with total hip arthroplasty, semi hip arthroplasty has the advantages of short operation time, less iatrogenic trauma, and fast recovery [5]. Therefore, it is the first choice for elderly patients who cannot tolerate major surgery and have good acetabula conditions on the affected side. At present, there are still some disputes about the fixation of femoral stem prosthesis. Due to the loss of calcium and phosphorus, the bone conditions of elderly patients are relatively poor [6]. In order to achieve satisfactory fixation effect in the early stage and enable patients to carry out weight-bearing exercise earlier, bone cement is chosen by more clinicians to fix the prosthesis stem. The use of bone cement can better adapt to the shape of the medullary cavity and provide a good early bite force between prosthesis and medullary cavity, so as to achieve a stable fixation effect and better restore patients' hip function [7]. However, the related complications brought by bone cement also limit its use to a certain extent, especially in elderly patients with poor cardiopulmonary function [8]. In addition, its long-term repair is more difficult. With the progress of biomedical technology, the development of biological prosthesis provides a new therapy idea for elderly patients with FNF. Exploring optimal strategies for the management of hemi hip replacement for elderly patients with FNF is of great significance for improving their quality of life and prognosis.

Hydroxyapatite (HA) is the main inorganic component of bone tissue, which has good bone induction and bone conduction, thus being more conducive to the formation of new bone [9]. Otherwise, its physical and chemical properties are significantly related to the particle size [10]. Compared with HA, the nanopore mechanism of nanoHA (nHA) can provide a larger contact surface area, thus providing a better scaffold for the adhesion and proliferation of osteoblasts [11]. In addition, because the nanostructure of nHA is conducive to the catabolism of osteoclasts, it has better biodegradability in vivo [12]. The biological prosthesis stem is coated with nHA, which is conducive to better promote the proliferation and adhesion of bone cells after implantation into the medullary cavity, thus improving its initial stability [13]. At the same time, the nHA coating on the surface of the prosthesis stem can make the medullary cavity completely closed, so as to provide good mechanical fixation [14]. In addition, in order to further promote the formation of new bone after biological prosthesis implantation, so as to obtain firm fixation, we applied platelet-rich plasma (PRP) to the therapy of FNF. Because PRP is centrifuged from autologous plasma, it has a large number of growth factors [15]. These growth factors are conducive to promote the proliferation of bone cells, and the formation of new bone after the prosthesis stem is implanted into the medullary cavity, so as to restore bone mineral density and better improve the initial stability of the prosthesis [16]. However, there are differences on the early fixation effect of biological prosthesis in FNF therapy in the elderly Therefore, in order to further explore the curative effect of cemented and biological prosthesis in the therapy of elderly FNF, we conducted research and discussion, and the results are as follows.

## 2. Materials and Methods

### 2.1. The Choice of Research Object

102 patients with FNF treated in our hospital from September 2018 to September 2021 were chosen as the subject investigated. Inclusion criteria are as follows: (1) clinical symptoms and imaging examination were consistent with the diagnosis of FNF, (2) unilateral fracture and initial hip replacement, (3) age range: 60–80 years old, (4) good limb movement function before fracture, (5) type Garden III and Garden IV, and (6) the expected life cycle is more than half a year. Exclusion criteria are as follows: (1) combined with other parts of bone fracture, (2) combined with metastatic malignant tumor, especially in hips, (3) unable to tolerate surgery, and (4) complicated with hip infection on the affected side. The above patients were randomly divided into bone cement group and observation group. All patients who participated in the study gave informed consent to the study and voluntarily signed informed consent. In addition, the study has been approved by the hospital ethics committee.

### 2.2. Preparation of PRP

Before operation, 60 mL venous blood was extracted and PRP was obtained by a two-step centrifugation. After centrifuging the venous blood samples at 1000 rpm for 10 minutes, the upper supernatant was collected and centrifuged again at 1000 rpm for another 10 minutes, and then, the light yellow supernatant suspended in the upper layer was removed to obtain the deposited PRP. The prepared PRP was placed on the rocking instrument for standby to prevent platelet coagulation.

### 2.3. Surgical Therapy

Bone cement group (*n* = 51): continuous epidural anesthesia is adopted, and the patient is in a healthy lateral position. After disinfection and towel lying of the operation area, improved Hardinge lateral incision is taken to cut the skin and subcutaneous muscle tissue in turn, so as to fully expose the joint capsule. Then, part of the joint capsule is cut to remove the femoral head, and the femoral neck is osteotomized. Medullary cavity is gradually expanded by medullary cavity drill and inserted the medullary cavity plug. After the bone marrow cement is filled with bone cement, suitable cement bone prosthesis (VerSys Advocate, Zimmer, USA) is placed, and then, the forward tilt angle of the prosthesis is adjusted before the cement is completely solidified. At last, the femoral head prosthesis is installed and the dislocation hip joint is reset. After checking the mobility and tightness of the hip joint, the drainage tube is placed, and the tissue at the incision layer is stitched by layer.

Observation group (*n* = 51): after the same operator exposed and cut the joint capsule in the same way as the bone cement group, the femoral neck is osteotomized and the medullary cavity is gradually expanded with a medullary cavity pressing file, and attention should be paid to the preservation of cancellous bone. After PRP is injected into the medullary cavity and applied on the surface of the biological prosthesis stem, the biological prosthesis (Corail, Johnson&Johnson, USA) is firmly embedded into the bone marrow cavity (Figure 1). At last, the anteversion angle is checked and appropriate bipolar femoral head prosthesis is installed. After the mobility and tightness of the hip joint are checked, the drainage tube is placed, and the tissue at the incision is sutured layer by layer.

### 2.4. Biological Activity Detection of nHA and PRP

Osteoblasts (CP-H111, Procell, Wuhan, China) will be cultured in 24-well plates for 24 h with complete culture medium for human osteoblasts (CM-H111, Procell, Wuhan, China) in cell incubator (51032124, Thermo Fisher, MA, USA) under 5% CO_2_ and 37°C, and then, these cells were collected and diluted with a PBS solution at a concentration of 1 × 10^4^ cells/mL. The above osteoblast diluents were divided into control group, nHA group, and NHA+RPR group. 1 mL osteoblast diluent and 2 mL special culture medium for human osteoblasts were added to each group, among which the control group was given no therapy, nHA sterilized by a high-pressure pot was added to the nHA group, and nHA and PRP were added to the nHA+RPR group. At last, the above cells were placed in the cell incubator and cultured for another 12 hours. Proliferation test will be performed by immunofluorescence. Anti-ki67 (ab15580, Abcam, USA) was used for labeling of living cells, and Alexa Fluor 488 (Cy2, FITC) was used as fluorescent secondary antibody. After incubation in dark at 26°C for 40 minutes, labeled cells were analyzed under a confocal microscopy (FV3000, OLYMPUS, Japan).

### 2.5. Detection of ALP Activity in Cultured Osteoblasts

The osteoblasts cultured in 2.4 were used to test mineralization ability. After the original culture medium was removed, cells were washed with a phosphate-buffered saline (PBS) solution for 3 times, and then, 200 *μ*L cell lysis reagent (C2360, Sigma-Aldrich, Merck, Germany) was added. The lysed cell liquid was placed in the alkaline phosphatase (ALP) detection board and used to detect the ALP activity. The detection process was strictly followed according to the detection method of ALP assay kit (ab83369, Abcam), and ALP activity was detected at 520 nm wavelength. In addition, PBS solution was used as blank control.

### 2.6. Detection of Bone Metabolism Level

In elderly fracture patients, the osteogenic ability and osteoclast activity have a key impact on the prognosis of fracture. In this study, bone alkaline phosphatase (BALP) and bone Gla protein (BGP) were used to reflect the ability of patients' osteoblasts, and procollagen type I carboxy terminal peptide (PICP) was used to reflect the activity of osteoclasts. 5 mL venous blood sample was collected before operation and at 2nd, 4th, and 6th week after operation. After centrifugation at 1000 rpm, the supernatant was taken. BALP enzyme-linked immunosorbent assay (ELISA) kit (Bke8846, Shanghai Boke Biotechnology Co., Ltd., China), human osteocalcin ELISA kit (ab270202, Abcam), and human PICP ELISA kit (EK-2076, Linyi Azeroth Biotechnology Co., Ltd., Shandong, China) were used to detect BALP, BGP, and PICP level in serum.

### 2.7. Evaluation of Clinical Therapy

The clinical recovery of patients was evaluated from the aspects of intraoperative bleeding, operation time, hospital stay, 48 h drainage flow, partial weight-bearing time, and complete weight-bearing time of affected limbs.

### 2.8. Comparison of Adverse Reactions

The adverse reactions were recorded, including periprosthetic femoral fracture, deep venous thrombosis, bone cement crisis, postoperative hip dislocation, pulmonary infection, and joint subsidence.

### 2.9. Comparison of Functional Rehabilitation and Life Quality

Harris score scale was used to evaluate the rehabilitation of patients' hip function in terms of pain, activity function, deformity, and range of motion [17]. In terms of life quality, orthopedic quality of life questionnaire (SF-36) [18] was used for evaluation. The questionnaire includes physical function, emotional function, role function, social function, and other dimensions. The score range of both scales was 0-100, and the higher the score, the better the corresponding hip function and life quality.

### 2.10. Statistical Methods

Statistical analysis and image rendering were performed on the data through SPSS 19.0 (Asia Analytics formerly SPSS China). The enumeration data were expressed by the number of cases/percentage (*n*/%), and the *χ*^2^ test was used to compare the data between groups. The measurement data were expressed as the mean ± SEM; the intergroup comparison was performed by independent samples *t*-test, the multigroup comparison was made by one-way ANOVA, and the intragroup comparison before and after treatment was performed by a paired *t*-test. When *P* < 0.05, the difference was statistically significant.

## 3. Results

### 3.1. Proliferation and ALP Activity Evaluation of Osteoblasts in Different Groups

The proliferation and activity of osteoblasts were important indicators to evaluate bone healing [19]. In this study, we evaluated osteoblast promotion states by fluorescence staining, and the brightness and range of fluorescence staining in the nHA group and nHA+PRP group were higher, especially in the nHA+PRP group (Figures 2(a)–2(c)). ALP was a marker of osteoblast mineralization function, and its activity could be used to evaluate the differentiation degree and osteogenic function of osteoblasts. Compared with the control group, ALP activity in the group added nHA and PRP was higher, especially in the nHA+PRP group (Figure 2(d)). These results suggest that biological prosthesis combined with PRP could promote the osteoblast proliferation, increase their activity, and promote bone healing.

### 3.2. Comparison of Bone Metabolism Level in Patients after Therapy

BALP, BGP, and PICP are important indicators often used to reflect bone formation in clinic [20]. Among which, BALP can reflect the osteogenic activity of osteoblasts, BGP is an important index of bone formation rate, and PICP can reflect the function of osteoclasts [21]. The study found that the levels of serum BALP and BGP in both groups reached the peak at fourth week after operation and then decreased slowly. The levels of the above indexes in the observation group were higher than those in the bone cement group (Figures 3(a) and 3(b)), suggesting that nHA and PRP can significantly promote bone formation and better maintain the stability of hip joint. However, the level of PICP increased gradually after operation, and it reached the highest at the fourth week, and then decreased gradually. PICP level in the observation group was lower than that in the bone cement group (Figure 3(c)), suggesting that nHA and PRP can reduce the activity of osteoclasts and reduce the rate of bone transformation, so as to promote the formation of new bone around the prosthesis.

### 3.3. Evaluation of Hospital Therapy in FNF Patients

In the study, patients' clinical therapy was evaluated from the aspects of intraoperative bleeding, operation time, hospital stay, 48 h drainage, partial weight-bearing time, and complete weight-bearing time of affected limbs. No significant difference was found between two groups (Figure 4), suggesting that the use of biological prosthesis combined with PRP can achieve the same stability as bone cement prosthesis and will not increase the trauma and difficulty of operation, thus effectively promoting the rehabilitation of elderly patients.

### 3.4. The Incidence of Complications after Therapy

In the experiment, the incidence of adverse reactions after therapy was evaluated in terms of femoral periprosthetic fracture, deep venous thrombosis, bone cement crisis, postoperative hip dislocation, pulmonary infection, and joint subsidence. The study found that the total incidence of adverse reactions in the bone cement group was higher, especially periprosthetic femoral fracture and bone cement crisis (Figure 5), suggesting that the use of nHA biological prosthesis combined with PRP can better avoid the adverse reactions of bone cement prosthesis and effectively restore the function of hip joint.

### 3.5. Comparison of Hip Joint Function and Life Quality after Therapy

After therapy, the recovery indexes of hip joint function in terms of pain, activity function, deformity, and motion range in the observation group could be better improved at different time points (Figure 6(a)). In addition, SF-36 scores in the aspects of physical function, emotional function, role function, and social function were lower in the bone cement group at different time points (Figure 6(b)). The above results suggest that nHA biological prosthesis combined with PRP is helpful to restore the stability of hip joint and better improve patients' life quality.

## 4. Discussion

In the surgical therapy of FNF, it is of great significance to restore the stability of hip joint at early stage, so as to enable patients to carry out weight-bearing exercise earlier, thus reducing the occurrence of postoperative adverse complications [22]. Early weight-bearing exercise is of great significance to improve patients' life quality and their prognosis, especially in elderly patients [23]. In order to maintain the good stability of hip joint after operation, it is mainly to have a good matching degree between prosthesis stem and medullary cavity. At the same time, it is necessary to promote the formation of new bone around the prosthesis stem, so as to obtain long-term stability of hip joint [24]. At present, in FNF therapy of elderly patients, bone cement prosthesis is widely used in clinic to obtain good fixation effect. Because elderly patients with FNF are often complicated with osteoporosis, they have the characteristics of enhanced osteoclast capacity and insufficient osteogenic function [25]. Therefore, it will have an adverse impact on the early stability and long-term fixation after prosthesis implantation. The use of bone cement prosthesis can make the prosthesis and medullary cavity firmly stick together, and fill the gap between bone trabeculae, so as to achieve good mechanical stability [26]. However, due to cardiopulmonary function in elderly patients is often poor, the toxic reaction of bone cement is easy to induce cardiac arrest and sudden drop of blood pressure during operation, which limits its use to a certain extent [8]. In addition, after bone cement is solidified, it will destroy the toughness of local femur, which is easy to lead to later femoral fracture [27]. Therefore, the development of biological prosthesis provides a new choice for FNF therapy in the elderly.

In order to achieve a stable fixation effect, biological prosthesis stem should be tightly combined with bone tissue, and the formation of new bone should be promoted. The surface of biological prosthesis is covered with nHA, and its large specific surface area provides a good scaffold for the proliferation of osteoblasts, which can effectively improve the osteogenic ability of osteoblasts [28, 29]. Otherwise, in order to further improve the osteogenic ability of osteoblasts after biological prosthesis implantation, we added PRP, which is obtained from autologous plasma after double centrifugation. Various growth factors rich in PRP can be used as extracellular matrix to provide a good living environment for the proliferation of bone cells and further promote the secretion of extracellular matrix [30, 31]. At the same time, it can also promote the blood supply of bone cells, thus better promoting their proliferation [32]. In the culture experiment of osteoblasts, we found that the addition of nHA and PRP effectively promoted cells' proliferation activity, and the mineralization ability of osteoblasts was greatly improved, especially in the nHA+PRP group, which is of great significance for the formation of new bone at the prosthesis stem and increasing its stability, thus promoting the early weight-bearing rehabilitation of elderly patients with FNF. Lin et al. [33] reported that nHA type I collagen beads combined with PRP as bone replacement can effectively promote bone regeneration, which is consistent with our research results.

The implantation of prosthesis will affect the level of bone metabolism. In elderly patients, increasing osteoblast activity and reducing osteoclast capacity will be conducive to their recovery. The study found that at 1st month after operation, the PICP level reflecting osteoclast activity decreased more significantly in the observation group; on the contrary, the BALP and BGP levels reflecting osteogenic activity increased more significantly. It is suggested that the use of nHA biological prosthesis combined with PRP reduces bone conversion rate and can better promote the formation of new bone around the prosthesis stem, so as to achieve the same early stability as bone cement prosthesis. In the study of Al-Ahmady et al. [34], the application of nHA combined with platelet-rich fibrin (PRF) in alveolar cleft repair technology significantly promoted bone regeneration of alveolar cleft defects, similar to our findings. Therefore, compared with the bone cement group, the use of biological prosthesis does not increase the difficulty of surgical therapy and medical trauma and can achieve the same early stability, so as to restore hip function and patient's early weight-bearing ability. Biomaterial-based augmentation techniques are also known to improve fracture stability and bone healing, with applications in the femur, tibia, proximal humerus, and distal radius [35]. In addition, the use of biological prosthesis effectively avoids the toxic effect of bone cement and the reduction of femoral segment compliance after adding bone cement, which can effectively avoid the occurrence of bone cement crisis and periprosthetic femoral fracture, so as to effectively reduce the incidence of postoperative adverse reactions, better restore hip function, and improve patients' life quality.

This study is novel in several aspects. First, it was confirmed from the aspects of osteoblast proliferation, ALP activity, and bone metabolism that the combined application of bioprosthesis and PRP can not only promote bone healing but also reduce the activity of osteoclasts to promote the formation of new bone around the prosthesis. Second, the efficacy and safety of nHA bioprosthesis combined with PRP in patients with FNF were confirmed from the perspectives of hospitalization, incidence of complications, hip function, and quality of life.

## 5. Conclusion

In this study, we explored the effect of nHA biological prosthesis combined with PRP in the therapy of elderly patients with FNF. We found that nHA combined with PRP could better promote the proliferation of osteoblasts and improve their mineralization ability, which is conducive to the formation of new bone after biological prosthesis is implanted into the bone marrow cavity, thus better restoring the early stability of hip joint. Compared with bone cement prosthesis, the use of biological prosthesis did not increase the difficulty of operation and iatrogenic trauma, but the same stability can be achieved, so as to better promote the early recovery of weight-bearing ability and reduce the complications caused by long-term bed rest. In addition, the use of biological prosthesis can effectively avoid the occurrence of bone cement crisis and periprosthetic femoral fracture, so as to better restore the function of hip joint and improve life quality. Therefore, the use of nHA biological prosthesis combined with PRP has its unique advantages in FNF therapy of the elderly.

## Figures and Tables

**Figure 1:** Action mechanism of nHA biological prosthesis combined with RPR.

**Figure 2:** Proliferative activity of osteoblasts in different groups. (a) Fluorescence of osteoblasts without any treatment. (b) Fluorescence of osteoblasts added nHA. (c) Fluorescence of osteoblasts added nHA and PRP. (d) Quantitative evaluation of ALP relative activity. ^∗^*P* < 0.05 and ^∗∗^*P* < 0.01.

**Figure 3:** Comparison of bone metabolism in both groups. (a) Changes of BALP level in the blood. (b) Changes of BGP level in serum. (c) Changes of PICP level in serum. Compared with that before operation, ^∗^*P* < 0.05.

**Figure 4:** Comparison of clinical treatment indicators between the two groups of patients. (a) Intraoperative bleeding and 48 h drainage volume. (b) Operation time, hospital stay, and partial and full weight-bearing time. ^#^*P* > 0.05.

**Figure 5:** Comparison of adverse reactions between two groups. (a) Adverse reactions in the bone cement group. (b) Adverse reactions in the observation group.

**Figure 6:** Comparison of rehabilitation between two groups. (a) Comparison of Harris score at different time points. (b) Comparison of SF-36 score at different time points. ^#^*P* > 0.05 and ^∗∗^*P* < 0.01.

## Data Availability

The labeled datasets used to support the findings of this study are available from the corresponding author upon request.
